This article has been retracted.

# An Optical Fiber Sensing Method for Measuring the Surface Flatness of an Object

**DOI:** 10.1155/2022/8023271

**Published:** 2022-06-27

**Authors:** Weijia Zhang, Qiancheng Rao, Zhenjie Gu, Peng Jiang

**Affiliations:** ^1^College of Electronic Information and Automation, Tianjin University of Science and Technology, Tianjin 300457, China; ^2^Tianjin Motimo Membrane Technology Co., Ltd., Tianjin 300457, China

## Abstract

Sensing of data or object is a mature research domain where intelligent devices, may possibly be embedded with the artificial intelligence-based techniques, are placed in the closed vicinity of the object or phenomenon. This sensing activity becomes more complex if it is related to the measurements of an object which is required to be accurate and precise. In this paper, the reflection interference spectrum method is used to measure the flatness of the surface of the object. The thickness of the tested object is between 0.4 and 16 *μ*m. The optical fiber sensor is moved on the surface of the object, and the reflection spectrum of each point on the surface of the object is analyzed. The thickness of each point, and through the movement of the stepping motor, the thickness of different points on the object is continuously measured, so as to obtain the surface topography of the object. This method has no destructive effect on the surface of the object, has no lateral test range limitation, and has a simple test system structure, High test accuracy, and reliable test results.

## 1. Introduction

Sensing of data or object is a mature research domain where intelligent devices, which may possibly be embedded with the artificial intelligence-based techniques, are placed in the closed vicinity of the object or phenomenon. This sensing activity becomes more complex if it is related to the measurements of an object which is required to be accurate and precise. These measurements are becoming more and more valuable and challenging as further improvements in the Internet of this technology have been reported in the literature. Apart from the technological improvement, various tests have been improved that is the accuracy of the result is relatively higher than those which is used previously.

With the continuous improvement of test and measurement technology requirements, the development of precision test technology is changing with each passing day [1]. The test of surface microtopography is an important branch of precision measurement technology, which has been greatly developed in recent years. At present, surface flatness test the methods mainly include contact measurement and noncontact measurement, and their test accuracy has reached the subnanometer level [2].

Contact measuring devices or instruments like elliptical polarisation offer simple measurement principles and vivid physical representations, therefore they are popular, but their measurement findings are not always accurate. It is impacted not only by the contour of the measured surface but also by the geometry of the stylus and the tension at the measuring point, which can easily damage the film surface, making it unsuitable for soft film measurement [3–5].

Noncontact measurement has become popular due to its high measuring speed and lack of harm to the film surface. A piece of test equipment that combines a microscope with an interferometer is known as microscopic light interferometry. It can assess the tiny unevenness of an object's surface to determine the bending degree of interference fringes, but data processing is difficult. STMs (scanning tunnelling microscopes) and atomic force microscopes (AFMs) are key advancements in precision measuring technology. The measurement precision is exceptionally good, and their lateral and longitudinal resolutions can reach subnanometer levels. The disadvantage is that the film flatness of the surface is required to be high, so the scope of use is limited. Many domestic research institutions also use the intensity of the reflected and scattered light on the surface of the object to study the measurement method of the surface flatness of the optical fiber sensor [6–8]. The object discussed in this paper is The surface flatness test method belongs to noncontact measurement. Through the analysis of the interference spectrum of the reflected light on the surface of the object, the thickness of the film is obtained, and the microtopography of the surface of the object is measured with the stepper motor [9, 10].

In this paper, we are going to develop an optical fiber sensing method for measuring the object's flatness surface which is realized or implemented through reflection interference spectrum a well-known approach. For this purpose, an optical fiber sensor is moved onto the respective surface to ensure analysis of each and every point of the concerned object.

The remaining paper arrangements are subjected to the following items.

Initially, in Section 2, the principle of the tests has been described in detail both in the textual and graphical format along with a discussion on how these tests are carried out and what are the main feature for the test. The structure of the proposed system is presented in Section 3 of the paper along with its different parts or sections. Example Test Analysis is presented in Section 4 of the paper where various tests have been carried out to ensure and verify the effectiveness of the proposed scheme in resolving the concerned issue. Lastly, a summary of the whole paper is given in Section 5.

## 2. Test Principle

In this section, we are going to describe various tests which have been conducted at the time of experiments to verify whether the proposed approach works according to the expectations or not.  Figure 1 depicts the single-point film thickness test principle. The light source is a broadband white light. When light from a light source contacts a film with a thickness of and a refractive index of *n*, reflected beams are created on the top and lower surfaces of the film, respectively. The incident light strikes the film and is reflected at the air-film interface, forming the first reflected light beam with an intensity of *I*_1_. The incident light passes through the film and is reflected at the film-carrier contact, where it is transmitted. It is pumped into the air via the film-air contact, resulting in a second beam of reflected light. The light intensity is *I*_2_. The reflected light is transmitted to the spectrophotometer by the optical fiber. This test method requires that the surface of the film carrier should be relatively uniform and flat.

When the refractive index of the film is low, the reflection of light in the film is very weak, and the case of multiple reflections is basically not considered, and there will not be multiple beams of coherent light, so only the coherence of the twice reflected light needs to be considered. Since the film has a certain thickness, there is an optical path difference Δ between the first beam and the second beam reflected light, Δ = 2*nδ*cos*i*, *i* is the incident angle of the light, under the condition of near-vertical incidence, *i* is approximately 0°, so Δ ≈ 2n*δ*cos(0)=2n*δ*. Within the coherence length of white light, the existence of the optical path difference may cause light interference between the two reflected lights. According to the Fresnel reflection formula, the light intensity of the interference light is

(1) $$\begin{array}{c} I=I_{1}+I_{2}2{\left(I_{1}I_{2}\right)}^{1/2}\cos\left(\frac{2\pi \Delta }{\lambda }\right). \end{array}$$

Here, *λ* is the wavelength of the incident light. Since the intensities of *I*_1_ and *I*_2_ are similar, they can be approximately considered to be equal. Assuming *I*_1_+*I*_2_=*I*_*R*_, formula (1) can be simplified as follows:

(2) $$\begin{array}{c} I=2I_{R}\left(1+\cos\left(\frac{2\pi \Delta }{\lambda }\right)\right). \end{array}$$

Equation (2) indicates that there is a cosine connection between / and *I* for a given. When/ = 0.5, 1.0, 1.5,…, the extreme value of reflected light intensity may be reached. If and when the connection between *I* and in equation (2) is a cosinelike relationship when the initialization value of is in the order of microns; that is, the shape is extremely similar to cosine, but as the value of increases, the period of the signal broadens, as seen in Figure 2.

Using the wavelength values corresponding to two or more extreme points, the order and delta value at each extreme point can be calculated. First find the extreme points *a*, *b*, *c*, and *d* and obtain the extreme point Corresponding wavelength *λ*_*a*_, *λ*_*b*_,…, set the order at *a*, *b*,… to 2*m*, (2*m* − 1),… in turn, and the order decreases because 1/*λ* decreases with the increase of *λ*, so the order The numbers should be decreasing. The equations are as follows:

(3) $$\begin{array}{c} \frac{4\pi n\delta }{\lambda_{a}}=2m\pi , \end{array}$$

(4) $$\begin{array}{c} \frac{4\pi n\delta }{\lambda_{b}}=\left(2m-1\right)\pi . \end{array}$$

For a given value of *λ*_*a*_, *λ*_*b*_, the value of *δ* can be obtained by solving equations (3) and (4) in succession.

## 3. System Structure

In this section, the structure or design of the proposed system is developed for the sensing of object movements. In Section 3.1, the composition principle of the design has been reported.

### 3.1. Composition Principle

In order to measure the surface flatness, the design of the instrument is shown in Figure 3. The light source used in the system is a 5 W tungsten halogen white light source, the Y-type optical fiber is a quartz multimode fiber, and the step size of the stepping motor is 55 *μ*m. The optical fiber provides light the conduction channel, the connection between the optical fiber and the light source, and the spectrum analyzer adopts the international standard optical fiber special SMA905 connector.

### 3.2. Optical Path

The broadband white light emitted by the light source is transmitted through the Y-type fiber, vertically incident on the film and is reflected back by the air-film interface and the film-carrier interface in turn to form the above-mentioned two reflected beams. When the two reflected beams are reflected by the same fiber when returning, it enters the other branch of the Y-type fiber through the Y-type fiber coupler and finally enters the spectrum analyzer. The spectrum analyzer records the interference spectra of the two coherent beams in real time, and the spectral data are sent to the computer, and a series of data are carried out. Treatment. The air gap between the fiber and the film must be much larger than the coherence length of the light source, so as not to be uncertain whether the interference spectrum comes from the air film layer between the fiber and the film, and the two beams of reflected light from the upper and lower surfaces of the film are coherent. result.

### 3.3. Spectrum Analyzer

A spectrophotometer, an AC/DC (A/D) converter circuit, and a computer make up the spectrometer. The spectrophotometer is an Oceanop-tics S2000 spectrometer that combines a spectrophotometer and an A/D converter circuit from the United States. The spectrophotometer is equipped with, as indicated in Figure 4, it is a cross-symmetric horizontal imaging system. The A/D converter circuit's output is routed straight to the computer's serial port for data processing. The spectrophotometer's slit is 25 metres long and one thousand metres tall, the reflection grating density is 600 lines per millimetre, and the imaging device is a SonyILX511 2048-unit CCD (Charge Coupling Device). The sampling frequency of the A/D conversion circuit is 500 kHz, the resolution is 12 bits, and the entire system is an optical resolution greater than 1.4 nm.

### 3.4. System Calibration

The silicon substrate used in the integrated circuit was oxidized to obtain a dense film on the surface of the object. The thickness of four points on the film was measured with an ellipsometer, and then the test method introduced in this paper was used to test and contrast. The results obtained are shown in Table 1.

The test error does not exceed 2 nm, and the error type is random, as shown by the test results in Table 1. This finding is quite exact, given the instrument's optical resolution limitations. If the overall system's optical resolution is to be enhanced, the system hardware must be modified. When the density of the reflection grating is raised by one order of magnitude (1 200 lines/mm), the optical resolution of the total optical system may also be enhanced by one order of magnitude, resulting in a test accuracy of better than 0.7 nm.

## 4. Example Test Analysis

A uniform polystyrene film is made on an opaque substrate with a high degree of finish, the film is fixed on the stepper motor, the position of the optical fiber detection system is fixed, and the position of the film relative to the fiber head is changed. The *x* and *y* of the horizontal plane move the diaphragm to be tested in the direction, test with 50 *μ*m interval length, test the point data of 16 × 20, and test the surface flatness of the diaphragm surface as shown in Figure 5.

## 5. Conclusion

Sensing of data or object is a mature research domain where intelligent devices, which may possibly be embedded with the artificial intelligence-based techniques, are placed in the closed vicinity of the object or phenomenon. This sensing activity becomes more complex if it is related to the measurements of an object which is required to be accurate and precise. The surface microtopography tester proposed in this paper is a new flatness measurement method based on the interference principle of white light and measured according to the spectrum of the reflected light. This method has high test accuracy and can test any area (the size is not limited), and there is no damage to the surface of the film. Because the structure of the detection system and the method of data processing are simple and the measurement accuracy of the instrument mainly depends on the resolution of the spectrophotometer, the stability of the light source itself, the stability of the film itself, the flatness and transparency, as well as the uniform flatness of the film carrier, can also be tested in the case of weak reflected light intensity.

## Figures and Tables

**Figure 1:** Test principle.

**Figure 2:** Cosinelike relationship between *λ* and *I*.

**Figure 3:** Instrument design.

**Figure 4:** Cross symmetry horizontal imaging system.

**Figure 5:** Example test of surface flatness. (a) Original test pattern. (b) Smoother surface after cubic interpolation.

**Table 1:** Test results of thin films on object surfaces.

Test point	Ellipsometer test results (nm)	Actual test results (nm)	Error (nm)
1	1003.4	1004.1	−0.7
2	1018.4	1017.3	1.1
3	1022.7	1021.4	1.3
4	1009.6	1009.3	0.3

## Data Availability

The datasets used and analyzed during the current study are available from the corresponding author upon request.
